The article "Effects of Fufang Banmao Capsule Associated with Sorafenib on Liver Function, Immune Status, Quality of Life Improvement, and Survival in Patients with Advanced Hepatocellular Carcinoma: A Retrospective Cohort Study" was retracted in 2023. Reasons: unreliable results or conclusions; concerns about the data; concerns about the peer review; concerns about the citations.

# Effects of Fufang Banmao Capsule Associated with Sorafenib on Liver Function, Immune Status, Quality of Life Improvement, and Survival in Patients with Advanced Hepatocellular Carcinoma: A Retrospective Cohort Study

**DOI:** 10.1155/2022/6336107

**Published:** 2022-08-23

**Authors:** Xianghong Lai, Anmei Wang

**Affiliations:** Department of Integrated Chinese and Western Medicine Oncology, Hangzhou Cancer Hospital, Hangzhou 310002, China

## Abstract

**Objective:**

A case-control study was carried out to explore the influences of Fufang Banmao capsule (FBC) associated with sorafenib on liver function, immune status, life quality, and survival in patients with advanced hepatocellular carcinoma (HCC).

**Methods:**

During January 2019 to October 2021, in our hospital, the clinical data of 144 patients with advanced HCC treated were collected and measured retrospectively. The patients were cured with transcatheter arterial chemoembolization (TACE) in the control group, and the patients were cured with FBC associated with sorafenib in the observation group. The clinical effect, liver function index, humoral immunity index (IgG, IgM, and IgA), cellular immunity index (CD3, CD4, CD4/CD8, and CD8), tumor marker alpha-fetoprotein (AFP), carcinoembryonic antigen (CEA), carbohydrate antigen 199 (CA199), and life quality were compared before and after treatment.

**Results:**

Regarding the therapeutic effects, the observation group had CR4, PR 48, SD 18, and PD2; the total remission rate was 97.22%. There were 2 individuals with CR, 32 with PR, 22 with SD, and 16 with PD in the observation group. 77.79% of the total remissions occurred. The total remission rate in the observation group was higher, and the difference was statistically significant (*P* < 0.05). A comparison of liver function index levels before and after treatment was done. As a result of treatment, the levels of AST, ALT, and TBIL lessened. In addition, the levels of AST, ALT, and TBIL in the observation group were lower as well, and the difference was statistically significant (*P* < 0.05). In the control group, the levels of serum IgG, IgM, and IgA were lower after treatment than before treatment, but in the observation group, the levels were higher. Additionally, the levels of IgG, IgM, and IgA were higher, and the difference was statistically significant (*P* < 0.05). With regard to the cellular immune indexes, compared to those before treatment, the CD3, CD4 and CD4/CD8 of the patients in the control group were lower, CD8 was higher, while CD3, CD4, and CD4/CD8 in the observation group were higher, CD8 was lower, and the difference was statistically significant (*P* < 0.05). AFP and CA199 levels lessened after treatment in the control group, indicating that the markers were reducing tumor growth, and the difference was statistically significant (*P* < 0.05). The value of CEA lessened, and the difference was statistically significant (*P* < 0.05). There was a marked decrease in AFP, CEA, and CA199 serum levels in the observation group compared to those before treatment, and the difference was statistically significant (*P* < 0.05). After treatment, the contents of AFP, CEA, and CA199 in the observation group were lower, and the difference was statistically significant (*P* < 0.05). In terms of the life quality after treatment, 36 patients (50.00%) had augmented KPS score and 38 patients (52.78%) had augmented ZPS score in the observation group, which was noticeably higher compared to the control group, and the difference was statistically significant (*P* < 0.05). The progression-free survival (PFS) of the observation group was 31.67 months (95% confidence interval was 0.09657∼0.3019), and the PFS of the control group was 26.73 months (95% confidence interval was 3.313∼10.36). The PFS time of the observation group was noticeably longer, and the difference was statistically significant (*P* < 0.05).

**Conclusion:**

FBC associated with sorafenib can noticeably strengthen the clinical effect of patients with advanced HCC, enhance the liver function and immune function of patients with advanced HCC, accelerate the speed of rehabilitation and ease clinical symptoms, reduce the level of tumor markers, strengthen the quality of life, and prolong the survival time of patients.

## 1. Introduction

Hepatocellular carcinoma (HCC) is the most common malignant tumor in the world with an upward trend year by year. The number of people in China is the highest in the world. Cytoreductive surgery is not only the first choice for the treatment, but also one of the most effective methods [1, 2]. In 2008, there were 700 thousand new cases of HCC in the world, and the incidence rate was 16 trillion. The Asia-Pacific region has a high incidence of liver cancer. More than 75% of the global HCC patients are concentrated in the Asia-Pacific region, and most patients are related to hepatitis B virus (HBV) infection [3, 4]. HCC patients in China account for more than 50% of the entire Asia-Pacific region [5]. The incidence of liver cancer is 26.68/100000 in China (39.42/100000 for men and 13.6/for women), which is second only to lung cancer and ranks second to lung cancer [6, 7]. In these areas with high incidence of liver cancer, it is urgent to find an effective treatment.

At present, cytoreductive surgery of tumor is still the primary choice and the most effective treatment for liver cancer. With surgical resection of liver lesions, the 5-year survival rate of patients has reached 60%–70% [8]. However, less than 20% of the patients can be surgically resected. HCC is usually discovered at a late stage for most patients, such as intrahepatic diffuse implantation, vascular invasion, or distant organ metastasis; the effect of surgical treatment in these patients is poor. In addition, HCC is not sensitive to chemotherapy and radiotherapy. Therefore, the treatment of advanced HCC still lacks effective treatment, which is still a major problem.

The pathogenesis of HCC is extremely complex and still not clear. However, some studies have found that the pathogenic factors affecting HCC are closely related to the geographical environment [9]. Hepatitis virus infection is strongly connected to the development and occurrence of HCC in the Asia-Pacific region. About 70% of HCC patients have HBV infection and about 20% of patients have hepatitis C virus (HCV) infection [9, 10].

HCC is a malignant tumor with rich blood supply [10]. In December 2005, Sorafenib (trade name Nexavar) was permitted by the Food and Drug Administration (FDA) of the US as a first-line drug of cancer and it was listed in China the next year. So far, Sorafenib is still the only first-line drug approved by many countries around the world for unresectable advanced HCC [11, 12]. Sorafenib is an oral polykinase inhibitor that exerts its antitumor effect by suppressing tumor cell proliferation and angiogenesis. Intracellular signal transduction pathway Raf/MEK/ERK and extracellular VEGFR and PDGFR have been proved to be closely related to the occurrence of HCC. The latest study found that Sorafenib inhibits the expression of MMP-2 and Ki-67 by upregulating the expression of PS3 gene and inhibiting the expression of FoxM1 (ForkheadboxM1) gene, thus blocking the proliferation of HCC cells and invasion of surrounding organs [13, 14]. Sorafenib can interfere with the above cellular signal transduction pathways, play a direct antitumor role in inhibiting the activities of c-Raf (Raf-1) and B-Raf, and play a dual antitumor role in antagonizing VEGFR-1,2,3 inhibiting the formation of tumor-related neovascularization.

Traditional Chinese medicine (TCM) preparation, especially TCM injection, is a great achievement in the field of medicine in China. However, its safety and efficacy have been widely concerned by the medical community since it was developed and listed on the market [15]. There has been more research suggesting that the application of TCM can noticeably reduce the incidence of radiation therapy and chemotherapy side effects and can enhance the cellular immunity and patients' life quality. Several TCM preparations have a synergistic effect on chemotherapy, which can not only prolong the duration of patients' survival, but also reduce the risk of metastasis and recurrence. Moreover, daily chemotherapy can increase the objective efficiency of chemotherapy. The TCM Fufang Banmao capsule (FBC), which is composed of Mylabris, ginseng, astragalus, Acanthopanax senticosus, mulberry,*Scutellaria barbata*, Rhizoma Curcumae, *Cornus officinalis*, *Ligustrum lucidum*, bear bile powder, and licorice, has the effect of breaking blood stasis and attacking white blood cells and phagocytic sores. Studies have indicated that in addition to inhibiting the growth of stem cells and apoptosis liver cancer cells, cantharidin also has a strong toxic effect, causing organ poisoning as well as necrosis [15, 16]. During January 2019 to October 2021, in our hospital, this study focuses on 144 patients with advanced HCC treated, which are reported as follows.

## 2. Patients and Methods

### 2.1. General Information

During January 2019 to October 2021, in our hospital, the clinical data of 144 patients with advanced HCC treated were collected and measured retrospectively. For the control group, the patients received TACE, while for the observation group, they received FBC plus sorafenib. There were 30 to 75 years of age in the control group and 31 to 76 years of age in the observation group. The control group average age was 52.18 ± 2.54, while the observation group average age was 52.34 ± 8.61. The general data were not statistically noticeable (*P* ＞ 0.05). The Medical Ethics Association authorized this study, and all patients noticed informed consent forms.

Inclusion criteria include the following: (1) abdominal CT examination, a large amount of fluid in the abdominal cavity; (2) certain abilities for understanding, expressing themselves verbally, and writing are present in patients and their families; (3) take part in the study and sign the informed consent form voluntarily and follow the principle of randomization; and (4) patients without heart, liver, and kidney vital organ disorders.

Exclusion criteria include the following: (1) mental illness patients or family members, or those accepting treatment in connection with mental illness; (2) patients with serious organ diseases; (3) exclusion of patients with KPS <70; (4) exclusion of patients with endocrine and metabolic diseases, such as severe diabetes, hyperthyroidism, and cardio-cerebrovascular diseases; and (5) exclusion of patients with a history of external injury and major operation within 1 month before treatment.

### 2.2. Treatment Methods

In the control group, patients were cured with liver TACE regimen. Seldinger puncture method, positive digital subtraction angiography (DSA), was performed after successful puncture; the location, quantity, and size of the tumor were accurately located; the guide wire catheter was inserted into the tumor feeding artery; and cisplatin and epirubicin were infused. The drug dose was used according to the individual condition of the patient. After operation, the guide wire was withdrawn, and the intervention point was pressed to stop bleeding. In the observation group, the patients were cured with FBC associated with Sorafenib and FBC orally (Guizhou Yibai Pharmaceutical Co., Ltd., Chinese medicine Z52020238), 3 tablets per time, twice a day. Oral administration during the intermission of chemotherapy: Each cycle was taken continuously for 21 days for 2 cycles as a course of treatment. Sorafenib (German Bayer Pharmaceuticals, imported Drug Registration no.: H20110599) 400 mg/times, twice a day. The subjects took the drug continuously and were originally scheduled to stop or reduce the dose when the patient developed a disease or could not tolerate side effects during treatment. After stopping or reducing the dose of sorafenib, the unified mode of administration was restored after the symptoms of the patients were enhanced. During chemotherapy, patients were given routine stomach protection, liver protection, immunity enhancement drugs, and early nutritional support treatment. The curative effects were evaluated at the end of one course of treatment.

### 2.3. Observation Index

#### 2.3.1. Evaluation Standard of Curative Effect

The response assessment criteria in solid tumors (RECIST) were used as evaluation criteria, complete response (CR), partial response (PR), stable disease (SD), and progressive disease (PD) [17]. CR: No new lesions appeared after the lesions disappeared; PR: More than 30% less tumor diameter was measured in the trial phase compared with the baseline phase; SD: Between PR and PD; PD: A greater than 20% increase in maximum and minimum tumor diameters or the appearance of new lesions occurred as compared with the baseline phase. Objective response rate (ORR): ORR = (CR + PR)/total number∗100%. Disease control rate (DCR): DCR = (CR + PR + SD)/total population∗100%. A CT examination was performed on all patients before joining the group, and a final CT examination was conducted after the treatment had ended. The same researcher enhanced the baseline and tumor evaluation during the treatment period.

#### 2.3.2. Liver Function Index Level

Before and after treatment, fasting venous blood of 3 mL was harvested, centrifuged 10 min, 3000 r·min^−1^, serum was separated, and serum levels of glutamic oxaloacetic transaminase, glutamic pyruvic transaminase, and total bilirubin were examined by enzyme linked immunosorbent assay (ELISA) (Beckman Coulter Co., Ltd.).

#### 2.3.3. Immune Function Index Level

The levels of serum CD3+, CD4+, CD8+, and NK before and after treatment were determined by Attune NxT acoustic focused flow cytometry and its supporting reagents, and CD4+/CD8+ was measured. The levels of IgM, IgG, and IgA in serum were measured by immune turbidimetry. The kits are all produced by Redd Company of the United States, and the testing operations are conducted in terms of the standards of the instructions, controlling intrabatch differences <10% and interbatch differences <15%.

#### 2.3.4. Tumor Marker Level

The venous blood of 5 ml was taken before and after one course of treatment, and the blood vessels were collected in vacuum. At room temperature, 10 min was centrifuged with 4000 r/min, and the upper serum was taken for the determination of AFP, CEA, and CA199 in serum.

#### 2.3.5. Quality of Life Score

The quality of life was evaluated by functional status score (Karnofsky, KPS) and physical status score (Zubrod-ECOG-WHO, ZPS).

#### 2.3.6. Survival Follow-Up

Patients were followed up by outpatient clinic and telephone, and the progression-free survival (PFS) from the beginning of treatment to the time of tumor progression or death was calculated.

### 2.4. Statistical Analysis

In order to process data and create charts, SPSS 22.0 statistical software is used; measurement data are presented as mean ± standard deviation (*x* ± *s*), and *t*-tests are used for comparison; counting data is presented by the number of patients and rate (%), and comparison is done by *χ*^2^ test. Survival curves were measured by Kaplan–Meier methods, and multivariate analysis by logistic regression analysis; a statistical difference was observed, and *P* < 0.05 indicated that the difference between groups is statistically significant.

## 3. Results

### 3.1. Comparison of the Balance of Basic Data of Research Objects

Our first step was to compare the balance of basic data. The average age, body mass index, sex, age distribution, clinical stage, degree of differentiation, and metastasis site showed no noticeable difference, and the difference was statistically significant (*P* < 0.05). In Table 1, all data results are presented.

### 3.2. Comparison of Clinical Efficacy

We compared the therapeutic effects. In the observation group, there were CR4 (*n* = 48), PR (*n* = 48), SD (*n* = 18), and PD2 (*n* = 18). The total remission rate was 97.22%. In the control group, there were 2 individuals of CR, 32 of PR, 22 of SD, and 16 of PD. The total remission rate was 77.79%. The total remission rate of the observation group was higher, and the difference was statistically significant (*P* < 0.05). In Figure 1, all data results are presented.

### 3.3. Comparison of Liver Function Indexes

Before and after treatment, we compared the level of liver function index, with no noticeable difference before treatment, and the difference was statistically significant (*P* < 0.05). After treatment, the levels of AST, ALT, and TBIL lessened. Compared between the two groups, the levels of AST, ALT, and TBIL in the observation group were lower, and the difference was statistically significant (*P* < 0.05). In Table 2, all data results are presented.

### 3.4. Comparison of Humoral Immune Indexes before and after Treatment

Before and after treatment, we compared the level of humoral immunity, with no noticeable difference in the levels of IgG, IgM, and IgA before treatment, and the difference was statistically significant (*P* < 0.05). Compared to those before treatment, the serum levels of IgG, IgM, and IgA in the control group were lower, while in the observation group, they were higher, and in the observation group, they were higher compared to the control group, and the difference was statistically significant (*P* < 0.05). In Table 3, all data results are presented.

### 3.5. Comparison of Cellular Immune Indexes

We compared the cellular immune indexes. Before treatment, there was no noticeable difference in CD3, CD4, and CD4/CD8, and the difference was statistically significant (*P* < 0.05). After treatment, CD3, CD4, and CD4/CD8 in the control group lessened and CD8 augmented, while CD3, CD4, and CD4/CD8 in the observation group augmented, CD8 was lower than that before treatment, and CD3, CD4, and CD4/CD8 in the observation group were higher, while CD8 was lower, and the difference was statistically significant (*P* < 0.05). All results are indicated in Table 4.

### 3.6. Comparison of Tumor Markers

We compared the levels of tumor markers. There was no noticeable difference in serum AFP, CEA, and CA199 levels before treatment, and the difference was statistically significant (*P* < 0.05). After treatment, the contents of AFP and CA199 in the control group lessened compared with those before treatment, and the difference was statistically significant (*P* < 0.05). The value of CEA lessened, and the difference was statistically significant (*P* < 0.05). The serum levels of AFP, CEA, and CA199 in the observation group were noticeably lower than those before treatment, and the difference was statistically significant (*P* < 0.05). After treatment, the contents of AFP, CEA, and CA199 in the observation group were lower, and the difference was statistically significant (*P* < 0.05). In Table 5, all data results are presented.

### 3.7. Comparison of Life Quality after Treatment

We compared the life quality after treatment. There was no noticeable difference in the number of patients with augmented KPS and ZPS scores before treatment, and the difference was statistically significant (*P* < 0.05). After treatment, KPS score augmented in 36 individuals (50.00%) and ZPS score augmented in 38 (52.78%) in the observation group, which was noticeably higher, and the difference was statistically significant (*P* < 0.05). In Table 6, all data results are presented.

### 3.8. The Survival Follow-Up Outcome

We compared the outcome of survival follow-up. The PFS of the observation group was 31.67 months (95% CI 0.09657∼0.3019) and the control group PFS was 26.73 months (95% CI 3.313∼10.36). The progression-free survival time of the observation group was noticeably longer, and the difference was statistically significant (*P* < 0.05). In Figure 2, all data results are presented.

## 4. Discussion

HCC is a kind of liver malignant tumor derived from epithelial tissue, which is highly malignant and invasive. HCC is the most frequent type of primary liver cancer, accounting for 91.5%, and it ranks sixth among all types of cancers worldwide. HCC is the third in tumor-related deaths after lung and gastric cancers [18, 19]. However, how to treat liver cancer is difficult, and the prognosis is poor. The annual recurrence rate of surgical resection is high. Most patients are found at the late stage; thus, the treatment becomes more difficult, resulting in worse prognosis.

Sorafenib is an oral polykinase inhibitor to treat advanced unresectable liver cancer [20]. Sorafenib is so far the first and only systemically targeted drug approved by multiple national drug inspection authorities for advanced liver cancer [11]. Sorafenib inhibits hepatoma cell proliferation, metastasis, and tumor neovascularization mainly by inhibiting Raf-1 and a variety of tyrosine kinase receptors, including VEGFR-1/-2/-3, PDGFR-*β*, c-Kit, FLT-3, and RET. After the first oral administration of 400 mgbid sorafenib, the maximum plasma concentration (*C*_max_) was 2.3–3.0 *μ*g/ml, and the peak time was generally 1.0–12.3 hours. After continuous administration of sorafenib, the steady-state plasma concentration was reached in about 7 days [11, 21]. Sorafenib has high bioavailability; however, a high-fat diet can reduce the bioavailability of sorafenib by about 29%. Therefore, it is recommended that patients take sorafenib on an empty stomach or 2 hours after meals to ensure maximum absorption. The binding rate of sorafenib to human plasma protein was high, and the in vitro experiment showed that the binding rate of sorafenib to human plasma protein was 99.5%. Sorafenib is cleared through liver metabolism and bile excretion [21]. Sorafenib is oxidized and metabolized by cytochrome P459 (CYP3A4) in the liver, and then 15% of the oxidative metabolites bind to glucuronide under the action of uridine diphosphate glucanosyl transferase 1A9. Studies have indicated that after oral administration of 100 mg sorafenib, 77% are excreted through feces and 19% through urine [22]. The elimination half-life of sorafenib is longer, up to 20–27 hours. The clinical efficacy of sorafenib when treating HCC has been confirmed by two phase III, randomized, double-blind, controlled, two large phase II clinical studies [22, 23]. Both SHARP and Oriental confirmed that sorafenib was effective and accurate when treating patients with advanced HCC, and the adverse reactions were mild [23]. After that, Korean scholars reviewed and studied the efficacy of sorafenib when treating advanced HCC patients with extrahepatic metastasis. There exhibited a median survival time of 9.6 months and a median period when the disease progressed of 2.5 months. Some scholars conducted a similar retrospective study, showing that, after sorafenib treatment, the median survival time of advanced HCC patients was 9.9 months, and the median time of disease progression was 3.8 months [24]. People who benefit from sorafenib include those with multiple intrahepatic cancer foci, lymph node metastasis, vascular invasion, and extrahepatic distant organ metastasis [25]. Although the efficacy of sorafenib when treating late stage is noticeable, the emergence of drug resistance to sorafenib has become a major factor hindering the further prolongation of the overall survival time of patients. In addition, the side effects caused by sorafenib, HBV infection, liver background, and other factors caused the difference in the therapeutic effect of sorafenib. Taken together, all these studies have confirmed that sorafenib has a noticeable and positive effect on advanced HCC and can noticeably prolong the PFS time and total survival time of patients with advanced HCC. During the treatment process, the adverse reaction sorafenib is mild, tolerable without serious fatal reaction occurrence.

The common side effects of sorafenib are diarrhea, weight loss, skin reaction of hands and feet, hair loss, and hoarseness [25]. Most of them were mild adverse reactions of grade CTCAE1 or grade 2, which could be relieved after reduction or symptomatic treatment, and the fatal adverse reactions were very few. SHARP and Oriental studies did not report the fatal adverse reactions of sorafenib when treating advanced HCC [22, 23]. Zhang et al. found that basal concentrations of angiopoietin (Ang2) and vascular endothelial growth factor (VEGF) are independent predictors of survival and can evaluate the sensitivity of HCC patients to sorafenib [26]. However, this method is difficult to monitor and carry out in clinical work. Some studies have found that early hand and foot skin adverse reactions are an independent prognostic factor of survival, and diarrhea can also be used as a predictor of survival [26]. Hand and foot skin reactions and diarrhea are also the most common adverse reactions when treated by sorafenib.

The TCM FBC, which is composed of Mylabris, ginseng, astragalus, Acanthopanax senticosus, Sangleng, *Scutellaria barbata*, Rhizoma Curcumae, *Cornus officinalis*, *Ligustrum lucidum*, bear bile powder, and licorice, has the effect of breaking blood stasis and attacking white blood cells and phagocytic sores. Its main ingredients include Mylabris, which belongs to the southern large Mylabris or yellow-black small Mylabris of turniaceae insects, can break blood stasis, attack toxin and phagocytic sores, and has the effect of anticancer, increasing white blood cells, and immune enhancement. Some previous studies have indicated that cantharidin can inhibit the growth of stem cells and accelerate the apoptosis of liver cancer cells, but it also has a strong toxic effect, causing organ poisoning and even necrosis [26, 27]. Astragalus membranaceus, which belongs to the dried root of Astragalus mongolicus or Radix Astragali, a perennial plant of Leguminosae, has the effects of replenishing qi and promoting yang, benefiting the body, promoting water and detumescence, detoxification, and muscle formation. Cancer cells are sensitive to chemotherapy due to astragalus saponins, its main component, which inhibits their growth [27]. The study also found that total astragalus saponins can inhibit the proliferation of mouse hepatoma H22 tumor cells, and its mechanism may be relevant to the enhancement of immune function [28]. Ginseng, the dried root of Panax ginseng, a perennial herb of Araliaceae, has the effects of tonifying vital energy, spleen and lung, and invigorating the mind. It has been found that ginsenosides can effectively reverse the multidrug resistance of HCC cells, and its mechanism may be related to the decrease of MDR1 and P-gp expression. There are also research findings; ginseng can successfully enhance the immunity of patients with liver cancer and reduce the incidence of adverse reactions [29]. Acanthopanax senticosus, Sangleng, *Scutellaria barbata*, zedoary, *Cornus officinalis*, Ligustrum lucidum, bear bile powder, licorice, and other drugs also have the effects of heat-clearing and detoxification, breaking blood stasis, tonifying and tonifying qi, and can enhance the clinical effect of chemotherapy in patients with liver cancer. From the aspect of TCM theory, FBC has comprehensive prescription and reasonable compatibility. It can promote the pathogenesis of qi stagnation, blood stasis, phlegm coagulation and dampness toxin by breaking blood stasis, attacking toxin and phagocytic sores, so that the functions of viscera, qi and blood and body fluid can be restored, and the balance between good and evil of the body can be restored. Modern medicine believes that FBC can promote the body's nonspecific and specific immune function, strengthen the body's immune ability, noticeably increase the tumor inhibition rate, and resist leukopenia caused by chemotherapy.

In this study, FBC associated with sorafenib was effective when treating patients with advanced HCC. It was found that the total remission rate of the observation group was higher. The levels of AST, ALT, and TBIL in the observation group were lower. After treatment, the levels of IgG, IgM, and IgA in the observation group were higher and the levels of CD3, CD4, and CD4/CD8 in the observation group were higher, while CD8 was lower. After treatment, the contents of AFP, CEA, and CA199 in the observation group were lower. KPS score augmented in 36 (50.00%) and ZPS score augmented in 38 (52.78%) in the observation group, which was noticeably higher after treatment. The progression-free survival time in the observation group was noticeably longer. Our results have shown that FBC associated with sorafenib can effectively inhibit the proliferation of tumor cells, enhance the immunity of patients, prolong their survival time, and improve their life qualities. There are some limitations in this study. First, the sample size of this study is not large, and it is a single-center study, so bias is inevitable. In future research, we will carry out multicenter, large-sample prospective studies, or more valuable conclusions can be drawn.

Conclusively, FBC associated with sorafenib has good clinical effect on patients with advanced HCC, which can noticeably enhance the quality of life of patients with liver cancer, inhibit the proliferation of tumor cells, enhance immune function and liver function, and promote the survival rate. However, for the longer-term effect, further clinical observation and follow-up are needed.

## Figures and Tables

**Figure 1:** Comparison of clinical efficacy. The blue color refers to the observation group and the gray color refers to the control group.

**Figure 2:** Comparison of survival follow-up outcomes. The red line refers to the observation group and the blue line refers to the control group.

**Table 1:** Comparison of general balance between groups (%).

Related factors	Observation group (*n* = 72)	Control group (*n* = 72)	*t*/*χ*^2^	*P*
Average age (years)	52.34 ± 8.61	52.18 ± 2.54	0.151	＞0.05

Body mass index (kg/m^2^)	24.78 ± 2.33	23.69 ± 2.56	2.672	＞0.05

Gender			1.039	＞0.05
Male	40 (55.56)	46 (63.89)		
Female	32 (44.44)	26 (36.11)		

Age distribution			0.516	＞0.05
30∼44 years	18 (25.00)	16 (22.22)		
45∼59 years	22 (30.56)	26 (36.11)		
60∼75 years	32 (44.44)	30 (41.67)		

Clinical staging			0.113	＞0.05
III B period	40 (55.56)	42 (58.33)		
IV period	32 (44.44)	30 (41.67)		

Degree of differentiation			0.508	＞0.05
High differentiation	22 (30.56)	20 (27.78)		
Middle differentiation	40 (55.56)	44 (61.11)		
Low differentiation	10 (13.89)	8 (11.11)		

Transfer site			0.154	＞0.05
Lymph node	56 (77.78)	54 (75.00)		
Bone	16 (22.22)	18 (25.00)		

**Table 2:** Comparison of liver function indexes between groups ($\bar{x}\pm s$).

Grouping	*N*	AST (U/L)		ALT (U/L)		TBIL (*μ*mol/L)	
		Before treatment	After treatment	Before treatment	After treatment	Before treatment	After treatment
Observation group	72	85.36 ± 1.25	41.85 ± 1.04^a^	95.14 ± 1.32	54.48 ± 1.16^a^	102.43 ± 1.18	62.58 ± 1.07^a^
Control group	72	85.75 ± 1.43	58.12 ± 1.18^b^	95.48 ± 1.25	63.87 ± 1.04^b^	102.58 ± 1.12	74.66 ± 1.15^b^
*t*-value		1.742	87.772	1.587	51.142	0.782	65.255
*P*-value		＞0.05	＜0.05	＞0.05	＜0.05	＞0.05	＜0.05

*Note.* Compared to observation group before treatment, ^a^*P* < 0.05. Compared to control group before treatment, ^b^*P* < 0.05.

**Table 3:** Comparison of humoral immune indexes between groups ($\bar{x}\pm s$, g/L).

Grouping	*N*	IgA		IgM		IgG	
		Before treatment	After treatment	Before treatment	After treatment	Before treatment	After treatment
Observation group	72	2.53 ± 0.18	2.87 ± 0.23^a^	1.83 ± 0.16	2.27 ± 0.15^a^	14.66 ± 1.34	16.37 ± 1.25^a^
Control group	72	2.64 ± 0.26	2.23 ± 0.31^b^	1.82 ± 0.22	1.53 ± 0.21^b^	14.35 ± 1.46	11.24 ± 0.66^b^
*t*-value		2.952	14.069	0.312	24.331	1.327	30.795
*P*-value		＞0.05	＜0.05	＞0.05	＜0.05	＞0.05	＜0.05

*Note.* Compared to observation group before treatment, ^a^*P* < 0.05. Compared to control group before treatment, ^b^*P* < 0.05.

**Table 4:** Comparison of cellular immune indexes between groups ($\bar{x}\pm s$).

Grouping	*N*	CD4		CD8		CD3		CD4/CD8	
		Before treatment	After treatment	Before treatment	After treatment	Before treatment	After treatment	Before treatment	After treatment
Observation group	72	36.31 ± 3.38	40.85 ± 4.14^a^	28.45 ± 2.23	24.45 ± 2.67^a^	59.64 ± 4.35	65.58 ± 6.25^a^	1.23 ± 0.13	1.48 ± 0.12^a^
Control group	72	36.37 ± 3.76	31.45 ± 3.05^b^	28.23 ± 3.22	30.35 ± 2.83^b^	59.48 ± 4.17	56.23 ± 5.24^b^	1.21 ± 0.15	1.11 ± 0.15^b^
*t*-value		0.101	15.511	0.477	12.867	0.199	9.728	0.855	16.344
*P*-value		＞0.05	＜0.05	＞0.05	＜0.05	＞0.05	＜0.05	＞0.05	＜0.05

*Note.* Compared to observation group before treatment, ^a^*P* < 0.05. Compared to control group before treatment, ^b^*P* < 0.05.

**Table 5:** Comparison of tumor markers between groups ($\bar{x}\pm s$).

Grouping	*N*	AFP (pg/ml)		CEA (ng/L)		CA199 (ng/L)	
		Before treatment	After treatment	Before treatment	After treatment	Before treatment	After treatment
Observation group	72	197.08 ± 17.45	89.93 ± 10.24^a^	36.06 ± 6.15	19.78 ± 3.05^a^	86.54 ± 13.58	53.74 ± 9.28^a^
Control group	72	201.18 ± 18.03	95.31 ± 11.87^b^	35.58 ± 5.93	27.47 ± 3.41^b^	85.67 ± 14.13	72.84 ± 10.46^b^
*t*-value		1.387	2.912	0.477	14.263	0.377	11.590
*P*-value		＞0.05	＜0.05	＞0.05	＜0.05	＞0.05	＜0.05

*Note.* Compared to observation group before treatment, ^a^*P* < 0.05. Compared to control group before treatment, ^b^*P* < 0.05.

**Table 6:** Comparison of quality of life between groups (*n*/%).

Grouping	*N*	KPS			ZPS		
		Raise	Stable	Drop	Raise	Stable	Drop
Observation group	72	22 (30.56)	36 (50.00)	14 (19.44)	23 (31.94)	35 (48.61)	14 (19.44)
Control group	72	36 (50.00)	23 (31.94)	13 (18.06)	38 (52.78)	25 (34.72)	9 (12.50)
*t*-value		6.281			6.442		
*P*-value		＜0.05			＜0.05		

## Data Availability

The datasets used and analyzed during the current study are available from the corresponding author upon reasonable request.
